The article "Three-Dimensional Reconstruction Algorithm-Based Magnetic Resonance Imaging Evaluation of Biomechanical Changes in Articular Cartilage in Patients after Anterior Cruciate Ligament Reconstruction" was published in 2022. Journal: Comput Intell Neurosci.

# Three-Dimensional Reconstruction Algorithm-Based Magnetic Resonance Imaging Evaluation of Biomechanical Changes in Articular Cartilage in Patients after Anterior Cruciate Ligament Reconstruction

**DOI:** 10.1155/2022/8256450

**Published:** 2022-03-15

**Authors:** Lu He, Yanlin Li, Hong Yu, Xinyu Liao, Zhengliang Shi, Yajuan Li, Guoliang Wang

**Affiliations:** Department of Sports Medicine, First Affiliated Hospital of Kunming Medical University, Kunming 650032, Yunnan, China

## Abstract

This study aimed to investigate the evaluation of biomechanical changes in articular cartilage in patients after anterior cruciate ligament (ACL) reconstruction by magnetic resonance imaging (MRI) based on a three-dimensional (3D) finite element model. The data of 90 patients undergoing arthroscopic ACL reconstruction in the hospital were collected and divided into the stable group (54 cases) and the unstable group (36 cases). A load of up to 134N was applied to the 3D finite element model, and the kinematics of knee flexion at 0°, 30°, 60°, and 90° were examined. The tibial anteversion, tibial rotation, and ACL/graft tension were recorded in the 3D finite element model, which was randomly divided into the normal group (intact group, *n* = 30), the ACL rupture group (deficient group, *n* = 30), and the anatomical reconstruction group (anatomical group, *n* = 30). When the graft was fixed at 0°, the anterior tibial translation at 30°, 60°, and 90° in the anatomic group was 8–19% higher than the normal value under 134 N anterior load. The tibial internal rotation in the anatomic group was 18% and 28% higher than the normal value at 30° and 90°. When the graft was fixed at 30°, the anterior tibial translation at 60° and 90° of the anatomic group was 15% higher than the normal value. The tibial internal rotation at 90° of the anatomic group was 16% higher than the normal value, and the above differences had statistical significance (*P* < 0.05). MRI images were used to assess the bone tunnel angle, and the statistical analysis by the independent-samples *t*-test showed that there were significant differences in the bone tunnel angle between the stable group and the unstable group (*P* < 0.05). Currently, based on the 3D finite element model, MRI can accurately evaluate the postoperative effect of anatomical ACL reconstruction in the position, diameter, and angle of tibial and femoral bone tunnels, which can be applied to clinical promotion.

## 1. Introduction

An anterior cruciate ligament (ACL) injury is a common and serious sports injury. Improper treatment leads to functional instability of the knee joint and can cause a series of residual lesions and seriously affect the motor function of the knee joint [1–3]. Cartilage injury secondary to ACL rupture was significantly higher than that caused by meniscus injury alone. ACL rupture not only leads to anteroposterior instability and rotational instability of the joint, but current biomechanical studies showed that ACL rupture leads to increased left and right lateral displacement of the joint, which leads to abnormal movement in all directions of the joint and can lead to abnormal movement of the patellofemoral joint [4, 5]. Survey data show that the incidence of acute ACL rupture complicated with cartilage injury is 26%, while the incidence of old injury complicated with cartilage injury is 75% [6].

At present, there are many studies related to ACL injury. The most used physical examinations in the clinic include the Lachman test, axial displacement test, and anterior drawer test. The Lysholm score is used to evaluate the knee joint function. The above four examinations are used to comprehensively diagnose the stability of ACL. After ACL injury, X-ray or enhanced computed tomography (CT) examination is often used to evaluate the surgical results, but the effect is not ideal [7–9]. Magnetic resonance imaging (MRI) is an indispensable means of examination. MRI is basically popularized in China, and the diagnostic accuracy is relatively high. However, how to improve the reading level of MRI in the later stage is an urgent problem for doctors in related disciplines, especially those who have just entered the field of sports medicine [10].

Although articular cartilage biomechanics play a key role in the research progress of arthritis, previous studies on ACL reconstruction mainly focused on the changes in kinematics after ACL reconstruction and the changes in the tension of the graft, and only individual studies explored ACL injury and the changes in articular cartilage biomechanics by reconstruction [11–14]. Specific articular cartilage contact stress values can be obtained using stress sensors and computer model stress analysis. Three-dimensional (3D) finite element model divides the outline of bone and cartilage layer from MRI images, mainly including femur and cartilage layer, tibia and cartilage layer, and ligament of knee joint and meniscus. Bone is regarded as a rigid body, and linear elastic material is used to replace the articular cartilage layer [15]. Hu et al. [16] applied 1000 N axial pressure to the knee joint of cadavers and found that MRI images based on the 3D finite element model were convenient for measuring the articular cartilage contact stress of medial and lateral compartments when the knee joint was almost straightened during single-beam ACL reconstruction. Wan et al.'s [17] experimental study in vivo indicates that ACL reconstruction will lead to cartilage degeneration; Fukuda et al [18] reported that ACL reconstruction can improve the stability of knee joint, and MRI images based on the 3D finite element model can measure the graft tension and cartilage contact stress. The operation of cadaver experiment is complicated, and the biomechanics (kinematics, graft tension, and cartilage contact stress) of knee joint under different load conditions cannot be fully measured after ACL reconstruction. Therefore, this experiment uses the 3D finite element model of knee joint to simulate anterior cruciate ligament reconstruction and studies the influence of single anterior cruciate ligament reconstruction on articular cartilage contact stress under different loads.

In this study, 90 patients with ACL injury were selected. The 3D finite element model algorithm was innovatively combined with MRI images for follow-up evaluation of patients after ACL reconstruction to investigate the effect of single-bundle ACL reconstruction under different loads on articular cartilage contact stress.

## 2. Research Objects and Methods

### 2.1. Research Objects

The data of 90 patients who underwent arthroscopic ACL reconstruction in the hospital from May 2018 to August 2020 were collected. The age was 18–60 years, with an average of 41.5 ± 10.6 years. There were 52 males and 48 females. All patients met the following inclusion criteria. According to the clinical diagnosis, they were divided into the stable group (54 cases) and the unstable group (36 cases). There was no significant difference in age and gender between the two groups (*P* > 0.05), indicating comparability (Table 1). Two experienced orthopedic surgeons performed knee stability tests and clinical scores within 3 months after operation and before MRI examination. This study was approved by the medical ethics committee of the hospital. All the patients and their families understood the study and signed informed consent.

Inclusion criteria are as follows: (1) popliteal muscle autologous reconstruction was adopted, and absorbable screws were selected to squeeze and fix the inner segment of tibial tunnel, with the inner diameter of 7.0 mm; (2) the time and methods of functional rehabilitation exercise after patient's knee surgery are consistent; and (3) MRI examination was performed 3 months after patient's reconstruction.

Exclusion criteria are as follows: (1) preoperative medial and lateral collateral ligament tear or bone contusion seriously affecting the stability of the knee; (2) patients with other diseases affecting functional recovery after knee surgery; (3) patients complicated with other diseases, such as tumors, mental disorders, and metabolic disorders; (4) other postoperative causes leading to graft tear; and (5) patients underwent ACL reconstruction.

### 2.2. MRI Examination Method

MRI was performed to collect images of the knee joint. The patient was foot advanced, and the knee was held in extension at 15–20° of external rotation, and the patient was instructed to remain quiet and emotionally stable to avoid artifacts due to shaking (matrix: 320 × 256; field of view (FOV):180 mm × 180 mm; slice thickness: 4.00 mm; and slice spacing:0.5–1 mm). Conventional examination sequences included the following: coronal using fat-suppressed fast spin-echo T2-weighted images (TSE-T2WI) (time of repetition (TR) = 3200 ms, time of echo (TE) = 77 ms); oblique sagittal using spin-echo T1-weighted images (SE-T1WI) (TR = 450 ms, TE = 13 ms); and transverse using fat-suppressed fast spin-echo proton density-weighted images (TSE-PDWI) (TR = 3800 ms, TE = 14 ms).

The bone tunnel size of the study subjects was observed and measured by MRI images, and the changes in the bone tunnel size of patients with different grafts and patients with re-rupture after ACL reconstruction were recorded and counted.

### 2.3. Imaging Evaluation Criteria

Determination of the location of the bone tunnel: the coronal femoral tunnel is located at the outer and upper edges of the posterior margin of the intercondylar fossa, the left knee is in the direction of 1–2 o'clock, and the right knee is in the direction of 10–11 o'clock. The sagittal femoral tunnel is located at the posterior quarter of the cortical line at the top of the intercondylar notch. The posterior margin requires the preservation of 1–2 mm of cortical bone (Figure 1(a)).

Bone tunnel measurement: the tibial and femoral bone tunnels were divided into three parts in MRI images, namely, distal tibia bone tunnel, mid-end embryo bone tunnel, and proximal tibial bone tunnel; distal femoral bone tunnel, middle femoral bone tunnel, and proximal femoral bone tunnel. Then, the coronal and cross-sectional images containing tibial and femoral bone tunnels were obtained in MRI. On the coronal plane, the tibial and femoral bone tunnels were divided into three sections on average, and the cross sections of bone tunnels at six different positions were located on this plane. Then, the cross-sectional values of bone tunnels at this point were measured on the cross section (Figures 1(b) and 1(c)). The size of the bone tunnel in 6 different positions of each patient was measured 3 times, respectively, and the average value was taken as the size of the bone tunnel of the current patient, and the expansion rate or reduction rate compared at operation time of the bone tunnel drilled at this time was calculated.

### 2.4. Construction of 3D Finite Element Model

The 3D finite element model of knee joint includes ACL, posterior cruciate ligament (PCL), medial collateral ligament (MCL), and lateral collateral ligament (LCL). Since the MRI images cannot accurately locate the ligament points of the knee joint, the digital conversion system MicroScribe G2LX was used to directly locate the insertion area of each ligament on the femur and tibia of the body, with the accuracy of 0.2 mm. The shape of the femoral condyle and tibial plateau is positioned by the digital conversion system as the bone markers of the knee joint. The digital conversion system imported the spatial data of ligament insertion location and special bone markers into MSC/Patran software by matching special bone markers and fused them with the remaining knee joint model (Figure 2).

In the 3D finite element model of the knee joint, the functional beam is used to replace the above ligament. The ligament deformation equation is as follows:

(1) $$\begin{array}{c} D=\frac{\left(L-L_{0}\right)}{L_{0}}, \end{array}$$

where *L* refers to the length of ligament after deformation, *L*_0_ represents the reference length of the ligament; that is, the length of the 0 load is the length of the ligament beginning to withstand tension. A piecewise function is used to represent the force-deformation equation.

(2) $$\begin{array}{c} F=\left\{\begin{array}{cc} 0, & D<0,\\ \frac{\left(1/4\right)kD^{2}}{D_{L}}, & 0\leq D\leq 2D_{L},\\ k{\left(D-D\right)}_{L}, & D＞2D_{L}, \end{array}\right. \end{array}$$

where *k* represents the stiffness parameter, *D*_*L*_=0.03, indicating the relative deformation of ligament tension. When the ligament deformation is greater than 2*D*_*L*_, the force and deformation are linear. If the ligament deformation is less than or equal to 2*D*_*L*_, the force and deformation are a quadratic equation of ligament deformation.

### 2.5. Experimental Simulation and Data Statistics of Anatomic ACL Reconstruction

The ACL rupture was simulated by removing all ACL functional bundles in the 3D finite element model of the knee joint. A single-beam nonlinear spring was used to replace the original ACL to simulate anatomical single-beam ACL reconstruction. The graft is a bone-bin tendon-bone graft with a stiffness of 10 mm. In the anatomical single-bundle ACL reconstruction, two tunnels with a diameter of 10 mm were made according to the center of the original ACL in the tibial and femoral attachment sites. To simulate screw fixation, all grafts were fixed at the entrance area of femoral and tibial tunnels (Figure 3).

The intact cadaver knee joint was placed on the Kawasaki robot test system (Kawasaki, Japan) for in vitro experiments to determine the stiffness of ligament elements and meniscus spring. In this test, the knee joints of cadavers were loaded up to 134 N, with an increasing load of 26.8 N in the anterior-posterior direction. As high as 10 Nm, the kinematics of knee flexion at 0°, 30°, 60°, and 90° were detected by 2 Nm increasing tibial internal and external rotation torque Kawasaki robot system. Abaqus commercial software (Dassault Simula, the USA) was used to calculate the finite element model. The tibial anteversion, tibial rotation, and ACL/graft tension were recorded in the 3D finite element model, which was randomly divided into the normal group (intact group, *n* = 30), the ACL rupture group (deficient group, *n* = 30), and the anatomical reconstruction group (anatomical group, *n* = 30). Anterior tibial translation, internal tibial rotation, and ACL/graft force were recorded.

### 2.6. MRI Image Analysis and Processing

The radiographs were independently read by two experienced radiologists, and the positions of the femoral and tibial tunnels and the transverse diameter of the corresponding bone tunnels were marked and measured, respectively, without knowing the results of clinical knee function assessment. If two radiologists disagreed, they reached an agreement after communication.

### 2.7. Statistical Methods

In this study, SPSS 22.0 was used as the analysis statistical software for statistical analysis. Enumeration data were expressed as percentage (%), data conforming to normal distribution were expressed as $\left(\bar{x}\pm s\right)$, and two independent-samples *t*-tests were used to detect changes in tibial and femoral angles in the stable and unstable groups. *P* < 0.05 was considered statistically significant.

## 3. Results

### 3.1. Knee Biomechanics under Anterior Loading

When the graft was fixed at 0°, the anterior tibial translation of the knee joint in the intact and deficient groups increased from 0° to 30° under 134 N anterior load and then increased from 30° to 90°, but the value of the deficient group was about 33–40% greater than that of the normal knee joint. Except for 0°, the anterior tibial translation at other knee flexion angles of the anatomic group was higher than that of the intact group. The anterior tibial translation at 30°, 60°, and 90° was 6.2 mm, 6.5 mm, and 6.1 mm, respectively, which was 8–19% higher than the normal value. The difference was statistically significant (*P* < 0.05) (Figure 4(a)). When the graft was fixed at 30°, the anterior tibial translation at 0° of the anatomic group was 2.4 mm, which was 29.4% smaller than the normal value, and the difference had statistical significance (*P* < 0.05). The values of anterior tibial translation of 60° and 90° were 5.8 mm and 5.7 mm, respectively, which were about 15% greater than the normal value, and the difference was statistically significant (*P* < 0.05) (Figure 4(b)).

Tibial internal rotation was 16–44% greater in the deficient group than in the normal knee. When the graft was fixed at 0°, the tibial internal rotation in the anatomic group was 6.4 and 7.3 at 30° and 90°, respectively, which were 18% and 28% greater than the normal value, respectively, and the difference was statistically significant (*P* < 0.05) (Figure 5(a)). When the graft was fixed at 30°, the tibial internal rotation at 0° of the anatomic group was 2.2, which was 37% smaller than the normal value. However, the tibial internal rotation at 90° was 6.6, which was 16% greater than the normal value, and the difference was statistically significant (*P* < 0.05) (Figure 5(b)).

In the normal group, the ACL tension did not change much at each knee flexion angle. When the graft was fixed at 0°, the graft tension in the anatomic group was 43.8 N, 25.4 N, and 7.6 N at 30°, 60°, and 90°, respectively, which was lower than the normal value, and the difference was statistically significant (*P* < 0.05). When the graft was fixed at 30°, the graft tension in the anatomic group was 149.8 N at 0°, which was greater than the normal group value. It was 43.8 N and 21.5 N at 60° and 90°, respectively, which was smaller than the normal value, and the difference was statistically significant (*P* < 0.05) (Figure 6).

### 3.2. Diameter and Size of Bone Tunnel

During follow-up, 52 cases of bone tunnel increased and 48 cases decreased compared with those during operation. The average enlargement of bone tunnel was −11.25 ± 12.46%, of which 6 cases were reconstructed with allogeneic ACL. The average enlargement of bone tunnel was −12.5 ± 8.63%. At 24 months after operation, 1 case was transplanted ligament ruptured again at the tibial attachment point, and the bone tunnel was the largest at the proximal tibial site (Figure 7).

The transplanted ligament was ruptured at the tibial attachment point 24 months after surgery (A: the bone tunnel position was located, and the bone tunnel position was located using the positioning line (solid line in the figure) in the coronal image; B: the transverse diameter of the bone tunnel, and the transverse diameter of the bone tunnel at each position was measured to be 1.25 mm in the right transverse section).

### 3.3. Evaluation of Bone Tunnel Angle by MRI Images

The bone tunnel angle was evaluated using MRI images, and the statistical analysis was performed by the independent-samples *t*-test (*P* < 0.005). The difference in bone tunnel angle between the two groups was statistically significant (*P* < 0.05) (Table 2).

## 4. Discussion

The ACL is the key anterior stabilizing structure of the knee joint and can maintain more than 80% of the limiting force effect of the knee joint. ACL injury will lead to knee instability, resulting in long-term meniscus injury, articular cartilage injury and degeneration, and arthritis in severe cases [19]. Arthroscopic ACL reconstruction is currently recognized as the best diagnosis and treatment, and when its stable function plays a role, the abnormal activity of the knee joint generally disappears and gradually returns to normal sports.

In this study, a 3D finite element model was used to simulate anatomic ACL reconstruction and counted the biomechanical performance of the knee model under anterior loading. The results showed that when the graft was fixed at 0°, the anterior tibial translation was greater than the normal group value at 30° of knee flexion, while the cartilage contact stress was greater than the normal group value at 0° of knee flexion. When the graft was fixed at 30°, the anatomic group was accompanied by increased graft tension and cartilage contact stress at 0° of knee flexion. The research literature of Tashiro et al. [20] reported that anatomical anterior cruciate ligament reconstruction would increase the tibial forward movement from 60° to 90° and make the knee joint loose. Grassi et al. [21] reported that anatomical anterior cruciate ligament reconstruction would lead to an increase in tibial forward movement and a decrease in graft tension at 0°to 90° of knee joint, which is different from our simulation experiment of knee joint kinematics under forward load. The reason for the difference may be that anatomical anterior cruciate ligament reconstruction can partially restore the biomechanics of knee joint, but the articular cartilage contact stress cannot be completely restored. In addition, graft tension is related to knee joint kinematics and cartilage contact stress.

Bone tunnel problems are the main cause of failure in ACL reconstruction, and abnormal bone tunnel position can lead to damage of the graft and cause joint instability. If the tibial tunnel is too posterior, or if the femoral tunnel is located close to the midline of the intercondylar fossa apex, it is easy to cause vertical change in the graft and unstable movement of the affected knee joint. If the tibial tunnel is too anterior and outward, the graft is easy to impinge on the intercondylar fossa apex and lateral wall. Due to the influence of target distance and knee joint positioning factors, the diameter of bone tunnel determined by ordinary X-ray film is often lower than the actual value. Although CT can show the location, direction, and internal fixation of the bone tunnel in multiple directions, it cannot accurately show the correlation between the bone tunnel and surrounding soft tissues. Compared with the above two imaging methods, MRI based on the 3D finite element model can not only perform omnidirectional and multi-angle imaging, but also accurately display the trend of bone tunnel. In addition, MRI based on the 3D finite element model can well display the soft tissue contrast and better evaluate the healing condition of graft and bone tunnel, which is consistent with the research results of Lv et al. [22].

If the tunnel angle exceeds 35° on the sagittal MRI image of the femoral tunnel and the tunnel outlet position is close to the joint capsule, it will cause damage to the patellofemoral joint and surrounding soft tissues. If the tunnel angle on coronal MRI images of tibial tunnel is less than 25° or more than 35°, it is easy to lead to instability of fixation device, edema of bone tunnel wall, expansion of inner diameter, extrusion of graft, and finally graft fracture. The results of this study showed that the knee stability was different when the coronal and sagittal femoral and tibial tunnel angles were different; the knee stability was higher when the coronal and sagittal femoral tunnel angles were between 25°–35° and 20°–30°, respectively; and the knee stability was higher when the coronal and sagittal tibial tunnel angles were between 25°–35° and 60°–70°, respectively. This is in general agreement with the findings of Nguyen et al. [23].

## 5. Conclusion

In this study, 90 patients undergoing arthroscopic ACL reconstruction were selected as the study subjects, and MRI based on three-dimensional knee finite element model was used to follow up and evaluate the patients after ACL reconstruction. This study shows that the current anatomical ACL reconstruction can restore part of the articular cartilage contact stress; MRI in the tibial and femoral bone tunnel position, diameter size, and angle can accurately evaluate the postoperative outcome. The limitations of this study are that the interference of factors such as graft and tendon healing cannot be excluded, the study base is small, and the study rigor is relatively insufficient. This conclusion needs to be confirmed by larger sample size, longer term, and more comprehensive research. In conclusion, the clinician's choice of appropriate tunnel position and angle can improve the postoperative success rate of ACL reconstruction.

## Figures and Tables

**Figure 1:** Location and size of bone tunnel. *Note.* (a) The location of the tunnel origin: after the intersection of the line drawn along the posterior femoral cortex (red) and the line drawn along the top of the intercondylar notch (yellow); (b) positioning of the tunnel. In the coronal plane image, the positioning line (solid line in Figure 1) was used to locate the bone tunnel position; (c) the transverse diameter of bone tunnel. The size of the transverse diameter of the bone tunnel at each location was measured in the transverse plane.

**Figure 2:** Three-dimensional finite element model of knee joint (femur, tibia, patella, cartilage, ligament, and meniscus).

**Figure 3:** Tunnel position and graft position for anatomic ACL reconstruction. (a) Tunnel position and (b) graft position. *Note.* The center of both tunnels is at the center of the ACL insertion.

**Figure 4:** Anterior tibial translation in the three groups under anterior loading. (a) Graft fixed at 0° and (b) graft fixed at 30°. *Note.*^*∗*^ indicated significant differences compared with the anatomic group (*P* < 0.05).

**Figure 5:** Tibial internal rotation in the three groups under anterior loading. (a) Graft fixed at 0° and (b) graft fixed at 30°. *Note.*^*∗*^ indicates significant differences compared with the anatomic group (*P* < 0.05).

**Figure 6:** ACL/graft tension in the three groups under anterior loading. (a) Graft fixed at 0° and (b) graft fixed at 30°. *Note.* indicates significant differences compared with the anatomic group (*P* < 0.05).

**Figure 7:** A 56-year-old male patient with allogeneic ACL reconstruction.

**Table 1:** Clinical characteristics of two groups of patients (*n*, %).

		Stable group (*n* = 54)	Unstable group (*n* = 36)	*P*
Mean age (years)		43.2 ± 10.5	44.5 ± 9.8	>0.05
Gender	Male	31 (57.4%)	21 (58.3%)	>0.05
	Female	23 (42.6%)	15 (41.7%)	>0.05

**Table 2:** Comparison of bone tunnel angles.

	Position	Stable group (*n* = 54)	Unstable group (*n* = 36)	*t*	*P*
Tibia	Coronal position	28.43 ± 6.35°	22.45 ± 6.32°^*∗*^	2.564	0.001
	Sagittal position	63.37 ± 6.25°	58.34 ± 7.47°^*∗*^	2.983	0.032

Femur	Coronal position	33.73 ± 7.39°	40.43 ± 13.38°^*∗*^	2.568	0.018
	Sagittal position	27.46 ± 5.59°	33.46 ± 9.49°^*∗*^	2.641	0.045

*Note.* ^*∗*^ indicates significant differences compared with the stable group (*P* < 0.05).

## Data Availability

The data used to support the findings of this study are available from the corresponding author upon request.
